The article "The Construction of English Smart Classroom Teaching Mode Based on Deep Learning" was published in 2022. Journal: Comput Intell Neurosci.

# The Construction of English Smart Classroom Teaching Mode Based on Deep Learning

**DOI:** 10.1155/2022/9037010

**Published:** 2022-08-22

**Authors:** Jianing Niu, Yang Liu

**Affiliations:** ^1^School of Foreign Languages, Dalian Jiaotong University, Dalian 116028, Liaoning, China; ^2^Maritime History and Culture Research Center, Dalian Maritime University, Dalian 116026, Liaoning, China

## Abstract

Deep learning has an increasingly far-reaching impact on classroom teaching and is an important trend driving the application of educational technology in schools. In the traditional lecture-style teaching process, students are mostly in a passive listening and memorizing state. Simple memorization and repeated training have a certain hindering effect on promoting the transfer and application of the learner's knowledge, and it is not suitable to exert the learner's subjectivity. This research uses the current rapidly developing wireless communication technology to transmit data to the English teaching management platform, so as to realize the information exchange between the English classroom monitoring terminal and the English teaching management platform. The monitoring terminal of the system is mainly responsible for data collection of information, such as student campus card information, the location of the monitoring terminal, and terminal equipment parameters, and uses wireless communication information technology to upload it to the English teaching management platform according to the communication protocol agreed between the terminal and the platform, and the English teaching management platform can issue instructions to the monitoring terminal, so as to realize the control and management functions of the monitoring terminal. The design of the English teaching management platform of this system is a Web system designed based on B/S architecture. The interface of the system is diverse, and English teachers can easily view the monitoring data on the platform through this system. The main function of the English teaching management platform is to receive the data collected from the monitoring terminal, parse the information, and display the processing results to the English teacher in the form of a page. In order to facilitate the storage of data, MySQL database is used for the background data storage of the English teaching management platform. Through the design of the hardware terminal module and the development of the English teaching management platform, a deep learning-based English smart classroom management prototype system is realized.

## 1. Introduction

In the information age, new things emerge in an endless stream, and the requirements for learners' autonomous learning ability and critical thinking ability are getting higher and higher. With the development of information technology and the wave of intelligent technology, deep learning has received the attention and attention of scholars. Deep learning advocates learners to actively transfer what they have learned to solve complex problems in reality, which helps to improve learners' own critical thinking and knowledge construction. Under the background of educational informatization, due to the support of the Internet and information technology, a variety of teaching tools and teaching resources have emerged that are conducive to teaching construction, an important direction of inquiry in teaching practice. How to use effective methods to realize deep learning of learners has become one of the research hotspots in the field of education. The development of Internet technology provides more possibilities for innovation in various industries, and network media has become an important medium for information and knowledge dissemination. Teaching is no longer a matter of students being satisfied with the transmission and indoctrination of teachers, but a resonant exchange and knowledge sharing between teachers and students in the classroom. In this context, the traditional indoctrination teaching mode obviously no longer meets the needs of teaching, and it has a certain limiting effect on stimulating learners' ability to innovate and transfer knowledge. The emergence of a series of “smart models” such as smart campuses, smart classrooms, representing new opportunities and challenges for the development of college education. Among them, smart classrooms, as a new teaching model, implement digitalization and personalization in the entire teaching process. Implementing deep learning for learners provides new ideas. Improve the quality of teaching by integrating intelligent data analysis, information sharing, and technology application with the entire teaching process. Information technology has brought strong support for educational reform. With the emergence and development of rain English classrooms, online English learning spaces, and microlecture English resources, the English teaching mode has begun to shift from “teaching-oriented” to “learning-oriented.” In recent years, in order to realize the deep learning of learners, scholars in the field of education continue to carry out teaching practices of various teaching modes. In the development of educational informatization, the application of teaching tools and information technology to improve teaching is an inevitable trend of educational development. Smarter classrooms are more in line with the requirements of the times. Smarter teaching tools are used to better integrate teaching content and teaching methods into classrooms and cultivate students' higher-order thinking ability. As a new teaching mode, smart classroom provides a new way of inquiry for the realization of deep learning.

IoT technology can help English learners to learn in a personalized, dynamic, and collaborative manner to solve problems in English learning and to engage in knowledge acquisition and sharing interactively. In addition, the way of learning goes beyond the traditional English classroom, and students can get information from anywhere. In traditional English classrooms, the English teacher is the source of information, learners must stay in the same place and participate in the same activities at the same time, and teaching styles often place students in a passive role. In the smart classroom, students' access to information is no longer single, and they will not be in a passive state. A smart classroom is not only a physical space to connect objects (smartphones, tablets, RFID tags, etc.), but also a learning environment for learners to learn and solve English learning problems [1–8]. From the perspective of the construction of the Internet of Things, this research first uses the Internet of Things-related acquisition modules to perceive the English classroom environment, designs the acquisition module of the English smart classroom, and then encodes the collected data. The data is transmitted to the IoT platform through the IoT network, and the data is analyzed and processed, so that managers can easily see the collected information.

## 2. Related Work

With the development of the Internet and technology, new learning methods are constantly emerging, and smart learning has received more and more attention. The environment that learning relies on is more digital. Learning in a smart environment integrates learning activities, textbook materials, and even teachers and classmates. These changes have made users put forward higher requirements for learning experience. The learning experience design based on the smart environment demand becomes increasingly important. Research on learning experiences in smart environments has focused on the design of learning experiences [9].

The main feature of scholars' research on smarter classrooms is case evidence. Most of the related researches on smarter classrooms conduct research experiments through actual teaching cases to prove the effect and feasibility of the design. The original intention of the design is to focus on the all-round development of students and to promote the cultivation of students' abilities as the core. Kumara and WW and others conducted smart classroom teaching environment experiments for teachers and students and analyzed learners' experience through questionnaires to verify whether the designed evaluation system can improve the teaching system and promote students' learning. Lee et al. proposed that, with the development of information technology, it is necessary to be good at applying technology, integrate technology and methods to form smart classrooms, and make smart classrooms specific and sustainable. Lui and Slotta applied designed experiential immersion learning activities to simulation experiments in biology. Using technology to display all aspects and enhance the experience and perception, through this experiment of teaching cooperation, the students participating in this course have formed a complete system of understanding of biological disciplines. Jena conducted an investigation and research on the learning situation of the smarter classroom, taking Indian primary school students as the research object, and came to the conclusion through the analysis and summary of the scores that the smarter classroom has more advantages in teaching strategies, teachers' roles, and the use of teaching aids. Kumara and others believe that the development of technology provides more possibilities for human-computer interaction, and the integration of somatosensory technology and classroom teaching reflects its advantages. Students gain a sense of pleasure through efficient human-computer interaction, and the proposed evaluation system is verified through questionnaires. It has positive significance for the development of smart classroom learning [10, 11].

To sum up, the integration and development of the Internet and education have accelerated the construction of smart teaching, using the information technology means of the new era to push the concept and method of blended teaching to a wider range and promote the cutting-edge information technology (such as cloud computing, Mobile Internet, data mining, etc.) integrated into teaching scenarios and committed to providing data-based and intelligent information support for all teaching processes.

## 3. Key Technologies of the English Smarter Classroom Management System

### 3.1. Overall System Design

The design of smart classroom management system based on NB-IoT communication technology is mainly composed of two parts: classroom management terminal and monitoring system. In the classroom, the collected data is sent to the monitoring system through the NB-IoT communication module through the information collection module, and the system analyzes the data for the administrator to view. This system is mainly designed from two aspects: the first is the hardware design; that is, the monitoring terminal is designed, and various IoT modules are used to expand the Arduino development board to meet the needs of teaching management; the second is the monitoring system. Design: the system mainly processes the data uploaded by the monitoring terminal, and the processing results are displayed to the English teacher in the form of text or graphics.  Figure 1 is the structure diagram of the system. The English teaching terminal transmits the collected data to the platform server through the NB communication base station through the core network. The administrator can see the data processed by the system in the system. It is displayed on the system page, which is convenient for English managers to manage the English classroom [12–14].

#### 3.1.1. The Overall Design of the English Teaching Terminal

English teaching terminal relies on the Internet of Things platform and adopts the relevant modules of the Internet of Things to design. The data collected by the terminal will be uploaded to the English teaching management platform through the Internet of Things communication module, and the English teaching management platform will process the data in real time and display it on the page; the administrator can understand the situation of the classroom accurately in real time, which brings convenience to the management of the classroom. The monitoring terminal designed in this study mainly collects the campus card information of the students in the classroom, the location of the classroom, and the status of the equipment, then encodes the collected data, and transmits the collected information to the English teaching management through the NB-IoT network platform and processes data in real time. As shown in Figure 2, the main function of the power module is to provide stable voltage to other modules. Since the monitoring terminal needs to work for a long time, in order to make the terminal run stably, the selection of the power module is particularly important. The acquisition module has two basic functions in design: the acquisition module will receive the command data from the main control module, and according to the instructions of the main control module, the corresponding acquisition unit (RFID module or positioning module) will be assigned to work for data acquisition. The module converts the collected parameter data into processable electronic information and sends it to the main control module for processing. The main control module encodes the collected data and sends the data to the English teaching management platform by calling the communication module. In the whole monitoring terminal, the main control module is at the core position. First, it controls the acquisition module and sends acquisition commands to the acquisition module for data acquisition. The second is to encode the data collected by the acquisition module according to the specified communication protocol and finally control the NB-IoT communication module to send the encoded data to the server, and the server analyzes the data in real time to realize real-time monitoring by the monitoring terminal [15–18]. The main function of the communication module is to monitor the data communication between the terminal and the English teaching management platform, to send data to the English teaching management platform and to receive data from the English teaching management platform. The configuration function of the monitoring terminal can be realized.

#### 3.1.2. The Overall Design of the English Teaching Management Platform

A properly designed English teaching management platform can fully tap the internal connection between the data. The function of the English teaching management platform is mainly to analyze and display the data uploaded by the monitoring terminal, and the administrator can easily monitor the collected data. In order to facilitate the management of the monitoring terminal and the reporting of the classroom location, the system will configure the monitoring terminal so that the terminal can report the location to the English teaching management platform in real time.  Figure 3 is the basic workflow of the English teaching management platform. It can be seen that the English teaching management platform receives the data uploaded from the acquisition device and extracts the data according to the agreed protocol format. First, the location data of the device is extracted, and the map module is called to locate the device. Then extract the flag bit of the acquisition device. The flag bit is mainly divided into two states: the state where the flag bit is 0 indicates that the monitoring terminal is currently working normally, and each module of the device is operating normally according to the settings. The data is stored in the database and then the data analysis module is called to process the data; if the flag bit is not 0, this state indicates that there is an abnormal situation in the acquisition equipment, and the platform will notify the management personnel of the abnormal information in time, thereby reminding the management personnel to take care of the abnormality and deal with it accordingly. Not only can the English teaching management platform analyze and process the uploaded data, but managers with corresponding management authority can also set parameters for monitoring equipment, such as the collection range of monitoring equipment, data collection cycle, and other instructions. After the parameters are configured, the English teaching management platform will issue a configuration instruction, the communication module will transmit the received data to the main control module, and the main control module will execute the instructions to configure the terminal and will automatically communicate with the English teaching management platform after the terminal has updated the configuration [19, 20].

### 3.2. Key Technologies of NB-IoT

NB-IoT is a wireless access technology that is standardized in 3GPP and has excellent performance to support IoT devices. IoT technology has good application prospects in many fields, such as security, asset tracking, remote monitoring, metering (gas, water and electricity, etc.), and smart grids. This enables the superiority of the Internet of Things to be reflected. Features such as large connections and low cost will support communications in these fields. The currently widely used 2 G/3 G/4 G/5G communication technologies cannot fully meet this demand. The structure design of smart classroom can be divided into the following three levels, as shown in Figure 4 [21].

The structure design of the smart classroom is designed according to the design mode of the Internet of Things: the bottom perception layer is responsible for sensing external information, such as the collection of external information by various sensors; the middle network layer is responsible for information transmission. The layer processes the data information passed by the network layer. These three-layer structures cooperate with each other to enable the IoT to operate stably. The following are the specific functions of each layer.

#### 3.2.1. Perception Layer

The task of the bottom perception layer is to collect information. The design of this research is mainly to collect the campus card information and the latitude and longitude information of the terminal.

#### 3.2.2. Network Layer

The network layer plays the role of data handling. It mainly uses wireless transmission to transmit the data information collected by the perception layer through the network layer, so as to realize multichannel data transmission and forwarding. The smart classroom communication technology chooses NB-IoT technology, which is more suitable for IoT communication because of its low cost and high security.

#### 3.2.3. Application Layer

The top-level application layer is at the core of the three-layer architecture. The application layer analyzes and processes the data sent by the network layer, saves the processing results in the database, and can generate a visual interface according to requirements.

NB-IoT technology is developed from 4G LTE/evolved packet core network (EPC). NB-IoT technology has many advantages that other communication technologies do not have, such as high coverage, low power consumption, etc. This technology optimizes the 4G network architecture to a certain extent. There are the following two transmission optimization schemes: (1) Control plane optimization transmission scheme: This scheme performs IP data transmission between the terminal and MME (Mobility Management Entity). The signaling bearer mechanism is used in the network, and the nonaccess bearer provides a security mechanism. (2) User plane optimization transmission scheme: This scheme mainly optimizes the signaling transmission process, so that the terminal can also store the connection in the idle state. The context information of the bearer is entered, and the wireless connection and the core network connection can be quickly reestablished for data transmission in an idle state. The overall architecture of NB-IoT is shown in Figure 5.

## 4. English Smart Classroom Teaching System Design

### 4.1. Design of the Data Acquisition Module

#### 4.1.1. Selection of the Data Acquisition Module

In order to facilitate the deployment of the terminal, the data acquisition module adopts MF RC522 radio frequency identification chip and Arduino development board. RFID (Radio Frequency IDentification) is a communication technology that can identify specific targets and read and write related data through wireless signals. Commonly used are low frequency (125∼134.2 kHz), high frequency (13.56 MHz), ultra-high frequency, and microwave technology. Among them, RFID readers are mainly divided into two categories: mobile and fixed, mobile such as handheld readers, etc.; fixed such as community access control. The Arduino development platform is suitable for a variety of hardware development. Similar to various development platforms, such as the VC development platform, the platform integrates various library files for various hardware development. In the development of hardware, the Arduino development platform can call existing functions without operating registers, and the development process is very convenient. Because the Arduino development board has the characteristics of scalability and easy operation, this design uses the Arduino development board to develop the acquisition device [22].

#### 4.1.2. Hardware Design of the Data Acquisition Module

The design of this module mainly collects the information of the student campus card, uses the MF RC522 radio frequency identification module to read the campus card, and then connects the module to the Arduino development board to complete the design of the module. The RC522 module communicates with the Arduino development board in a synchronous serial manner. The Arduino development board and the RC522 module work separately. The connection between the module and the Arduino development board is shown in Figure 6.

### 4.2. Design of the Wireless Communication Module

#### 4.2.1. Selection of the Wireless Communication Module

In the design of the Internet of Things system, the selection of the appropriate communication module will have a huge impact on the overall stability of the Internet of Things. The stable and accurate transmission performance of the communication module provides a reliable guarantee for the transmission of the entire data. Therefore, in this design, the BC95 wireless communication module with excellent performance was finally selected. The communication module has the following advantages: (1) Small size: the monitoring terminal designed in this study is small in size, and the size of the communication module should match the size of the monitoring terminal. Therefore, the size of the module should be considered when selecting a wireless communication module. The BC95 module selected in this design has an area of about 4 cm^2^, which can meet the design requirements of the monitoring terminal. (2) Ultra-low power consumption: the module can run stably at ultra-low current, with a minimum current of 5 *μ*A. (3) LCC package: the use of LCC package can greatly increase its output, which is suitable for mass purchase. (4) Network characteristics: it can be compatible with most network protocols in terms of communication capabilities, which makes the application scenarios of this module more abundant. (5) Work wide temperature range: the highest temperature resistance can reach +85°C, and the minimum temperature resistance can reach −40°C, which enables the module to cope with various complex temperature environments. (6) AT (Attention) command: in order to facilitate the writing of programs, the module supports many AT commands, which will greatly reduce the workload of programming. From the above advantages, the BC95 communication module has excellent performance and a wide operating temperature range. It is an excellent NB-IoT wireless communication module. Its small size meets the small size requirements of the system design. At the same time, the packaging of BC95 is not difficult. LCC packaging method can be used, and SMT equipment can be used to achieve mass production, which can meet a large number of configurations of monitoring terminals. In order to enable the BC95 module to cope with various complex environments, the use of SMT, a difficult patch technology, enables the module to have good performance and high reliability.

By Figure 7, it can be seen that the BC95 module provides a large number of interfaces on the outside and also provides two data storage units, Flash and SRAM, inside the module. Data can be stored here, which can effectively prevent data loss. The module also supports an external USIM card to transmit data through the network provided by the USIM card. There is an external interface for the SPI communication module for data transmission, which is convenient for data transmission. The network frequency bands supported by the module are rich, and the sending and receiving modes of Band5, Band8, Band20, and Band28 are supported [23, 24].

#### 4.2.2. Circuit Design of the Wireless Communication Module

In order to reduce the energy consumption of the entire monitoring equipment, in the process of designing the communication module, it is necessary to ensure that it starts up during working hours and sleeps during nonworking hours, so as to reduce the overall energy consumption. The main control module will send a sleep command to the communication module, and the communication module will enter the sleep mode after receiving the command. When the main control module sends a power-on command again, the communication module will be awakened to perform normal data reception and transmission. The specific working time arrangement can be parameterized on the English teaching management platform.

Figure 8 is the pin diagram of the BC95 communication module. This module mainly uses the following pins: Pin 15 is reset, which is used to control the switching operation of the communication module. It can be directly connected to the development board by using a triode. The pin can detect whether the communication module is registered to the network, and the light-emitting state of the diode can be observed by connecting a triode to the light-emitting diode. The switch state of the light represents whether the module can be successfully registered to the network, as shown in Table 1.

Pins 29 and 30 are connected to the development board and are responsible for data transmission between the communication module and the development board. Pins 38–41 are used to connect the USIM card to provide mobile network services for the module, and pins 46 and 54 are for the communication module, providing power input interface. The 53-pin is connected to the external antenna, which increases the stability of the module signal and improves the ability of data transmission and reception.

### 4.3. Hardware Design of the Positioning Module

In this research design, the location of the monitoring terminal is also required to be located; the purpose is to be able to understand the distribution of the terminal and to find the equipment in time when the terminal equipment fails to reduce equipment maintenance costs. Since the monitoring equipment is distributed in all corners of the classroom, the positioning accuracy of the positioning module is required to be high. Selecting a suitable positioning module will be beneficial to the analysis of the data of the English teaching management platform and the maintenance of the equipment by the managers. At present, it can receive satellite signals of Beidou B1 frequency band and GPS frequency band and monitor the real-time location through the location acquisition of the positioning module.

#### 4.3.1. Selection of the Positioning Module

In order to achieve equipment positioning in indoor conditions, this study also has certain requirements for the power supply voltage of the module. The following is the parameter comparison between various module models.

By Table 2, it can be seen that the NEO-M8N positioning module has higher positioning accuracy than other models, and the smaller size of the module meets the requirements of the monitoring terminal module selection. After a variety of parameter comparisons, the NEO-M8N module is finally selected as the positioning module of the monitoring equipment. The NEO-M8N module has the following advantages: (1) It can receive 4 types of satellite signals at the same time, calculate the best positioning position according to the received satellite signals, and also provide high precision in some weak signal scenarios satellite positioning. (2) The navigation sensitivity is high, which is not the high sensitivity of other modules, reaching −167 dBm, which has good support for all satellite augmentation systems. (3) It has ultra-low energy consumption, and low power consumption does not mean a reduction in performance; on the contrary, the module performs well even at low power consumption, thanks to the support of an advanced architecture. The built-in energy-saving algorithm of the module can automatically optimize the power consumption of the module according to the actual scene. (4) Strong anti-interference ability: the module has a front-end LNA (Low Noise Amplifier) to achieve easier antenna integration and front-end SAW (Surface Acoustic Wave) filter, the anti-interference ability has been improved, and it can cope with most scenarios.  Table 3 is the performance parameters of NEO-M8N.

#### 4.3.2. Circuit Design of Positioning Module

The workflow of the positioning module is shown in Figure 9.

By Figure 9 it can be seen that the positioning module will automatically search for satellites and perform positioning when it is powered on. The position data after positioning will be sent to the development board through the serial port, and the position data will be encoded by the main control module and then uploaded to the English teaching management platform by the communication module. Realize the monitoring of the monitoring terminal position. After the positioning module sends data, in order to save power consumption, the positioning module will be turned off at this time.

As can be seen from Figure 10, the module's external ceramic antenna GPS1003 is connected to the positioning module through pin 11. Pins 21 and 20 are connected to the asynchronous serial port of the development board to provide data and output of data. Connect two capacitors and inductors at the 23 pin. The role of the inductor can effectively reduce the electromagnetic interference to the module and effectively improve the anti-interference ability of the positioning module. The two capacitors added to pin 23 mainly play the role of decoupling and increase the stability of the power supply of this pin. Pin 22 is the backup power pin, and the power supply is connected to it through a step-down diode and a capacitor. The advantage of this connection is that after the positioning module is accidently powered off in a short period of time, the module can be discharged through the capacitor, which can ensure that the device can work as quickly as possible. The location information can be obtained by using the Arduino development board to connect the positioning module. Since the ceramic antenna connected to the module has a strong GPS signal receiving ability, it also has a good effect in the classroom. In addition, the positioning module also provides time and speed. For this device, it is only necessary to obtain the latitude and longitude information of the device. The wiring diagram of the positioning module and the Arduino development board is shown in Figure 11.

## 5. Test of the English Smarter Classroom Teaching System

### 5.1. Function Test of the Data Acquisition Terminal

The function of the monitoring terminal is to collect student campus card data and terminal latitude and longitude information and upload it to the English teaching management platform through the communication module. This section will perform functional tests on the acquisition module and communication module to ensure the reliability of the monitoring terminal. When the function test of the acquisition module of the monitoring terminal is performed, the written acquisition program needs to be programmed into the development board. This test is mainly carried out by printing the data collected by the monitoring terminal to the PC screen through the serial port debugging tool, with data display.

#### 5.1.1. Data Acquisition Module Test

Before testing the data acquisition module, you first need to know what information is contained in the data uploaded by the monitoring terminal. In order to facilitate the analysis of the uploaded data and observe the results, because the use of the acquisition terminal by students is a random event. The student's campus card information is collected, so here it is judged whether the last two bytes are student information.

This test adopts the method of direct observation of the source data, and the data has not undergone secondary conversion in the format, which ensures the accuracy of the source data. The data in the data frame is decoded by the relevant software, and the decoded data is printed on the PC screen by means of printf resetting. In this test, the USR-TCP232 network debugging assistant is used to debug the data acquisition. Data will be collected at regular intervals, here the time interval is set to 5 seconds, and the data collection test chart is shown in Figure 12. In the process of testing the RFID module, the card reading operation is performed, and the data shows that the student information has changed. Through the movement of the data acquisition module, it can be observed that the position information transmitted by the serial port has changed, and its flag bit has also changed accordingly.

#### 5.1.2. Network Communication Function Test

Since the NB-IoT module needs to configure the selection parameters of the working mode before use, the CoAP mode is selected as the data transmission mode in the working mode, and the other transmission modes include the transparent transmission mode and the UDC mode. CoAP mode is a lightweight protocol that is very suitable for this small IoT terminal. The parameters of CoAP mode can be configured using AT commands. The main AT commands are shown in Table 4.

The working mode can be configured through AT + WKMOD, for example: AT + WKMOD = UDC means to switch the working mode to UDC mode, and similarly, it can also be switched to CoAP mode.

Before testing whether the communication module can successfully connect to the network, it is necessary to install the SIM card and connect the antenna. After making preparations, connect the module to the PC through the serial port and observe its communication. The data format is “AT + NMGS = number of bytes, data.” It can be seen from Figure 13 that after the communication module sends data, the server returns the data and prints “OK” through the serial port, which proves that the communication network is normal.

### 5.2. Data Analysis Module Test

For data statistics, the statistical data includes management summary table, attendance rate, alarm message, and classroom resource usage table, and the attendance statistics list viewing function is also provided in the upper right corner of the statistical analysis page, which is convenient for administrators to check the attendance status of students in the selected date range. Its interface is shown in Figure 14.

In the Figure 14, the user can clearly see the results of the data analysis. After the user selects the appropriate date on this interface, enters the correct class schedule, and selects the classroom and clicks the OK button, the system will automatically generate the corresponding chart according to the selection and generate corresponding student attendance statistics list.

## 6. Conclusion

In the process of the development of traditional education to modern education, information and communication technology has become an identification tool for modern people. It plays an important role in the teaching process and is more valuable than traditional peripheral devices. It is an important asset in learning. Among these innovative technologies, the Internet of Things is the main direction of innovation in various scenarios of our daily life, and it also has a good performance in education. It creates a new form of interaction between teachers and learners, which helps to improve the teaching process and create a relaxed and enjoyable learning environment for students. In this paper, combined with the actual needs of the smart classroom, the NB-IoT Internet of Things wireless communication technology is used as the communication method of the smart classroom management system to design the system. Select the classrooms in the campus as the carrier of the terminal monitoring node, collect the campus card information and the location information of the terminal at the same time, and upload the collected information to the English teaching management platform through the NB-IoT technology. The parameter configuration is realized by sending instructions to the terminal, so as to realize the remote real-time monitoring of the classroom and the functions of managing monitoring equipment. After long-term use in the future, the system will have a problem of large concurrency, which will cause the server to run slowly. Therefore, the overall performance of the system needs to be further optimized.

## Figures and Tables

**Figure 1:** English teaching system structure diagram.

**Figure 2:** Design of the monitoring terminal.

**Figure 3:** The workflow of the English teaching management platform.

**Figure 4:** Smart classroom structure design.

**Figure 5:** NB-IoT network architecture.

**Figure 6:** RFID module and Arduino module connection diagram.

**Figure 7:** BC95 function diagram.

**Figure 8:** BC95 communication module pin diagram.

**Figure 9:** NEO-M8N module workflow.

**Figure 10:** Peripheral circuit design of positioning module.

**Figure 11:** NEO-M8N wiring diagram.

**Figure 12:** Data acquisition test chart.

**Figure 13:** Network communication test chart.

**Figure 14:** The attendance status of students in the selected date range.

**Table 1:** Netlight and module working status.

Netlight status	Module working status
Lights off	Module registration network failed
Light	The module registered the network successfully

**Table 2:** Comparison of various models of modules.

Module model	NEO-M8N	UM220	BD-228	TM8620	MXTOS2-200
Operating voltage (V)	3.0–3.6	3.0–3.6	3.0–3.6	3.0–3.6	5
Positioning accuracy	Less than 3 m	3 m–5 m	Less than 5 m	Less than 10 m	3 m–5 m
Cold start time	About 25 s	About 35 s	About 34 s	About 38 s	About 37 s
Warm start time	About 3 s	About 1 s	About 6 s	About 1 s	About 2 s
Recapture time	Less than 1 s	Less than 1 s	Less than 1 s	Less than 1 s	Less than 1 s
Size (mm)	12.2 ∗1 6 ∗ 2.4	17 ∗ 22.4 ∗ 2.4	40 ∗ 30 ∗ 2.8	20.2 ∗ 40.7 ∗ 2.3	20.2 ∗ 40.7 ∗ 8

**Table 3:** NEO-M8N performance parameters.

Operating voltage	3.0–3.6 V	
Energy consumption	50 mW	
Sensitivity	Capture	−148 dBm
	Track	−165 dBm
Positioning accuracy	Less than 3 m	
Frequency	GPS, L1, 1575.2 MHz, C/A code	
Module size	12.2 *∗* 16 *∗* 2.4 mm	
Maximum refresh rate	10 Hz	

**Table 4:** AT commands in the CoAP mode.

AT command	Function description
AT + WKMOD	Work mode query/selection
AT + NPING	Query network connection
AT + NMGR	Read message
AT + NMGS	Send a message
AT + NSMI	Enable send notification
AT + S	Save the current running parameters
AT + Z	Restart the module
AT + CFUN	CoAP configuration temporary command switch
AT + NCDP	Set CoAP server address port

## Data Availability

The dataset can be accessed upon request to the corresponding author.
